The article "Diagnosis and Treatment of Vascular Surgery Related Infection" was retracted in 2018. Reason: compromised peer review.

# Diagnosis and Treatment of Vascular Surgery Related Infection

**DOI:** 10.2174/1874120701509010250

**Published:** 2015-09-17

**Authors:** Yong-Gan Zhang, Xue-Li Guo, Yan Song, Chao-Feng Miao, Chuang Zhang, Ning-Heng Chen

**Affiliations:** Department of Vascular Surgery, First Affiliated Hospital, Zhengzhou University, China

**Keywords:** Antibiotics, diagnosis, infection, treatment, vascular surgery

## Abstract

Surgical site infection (SSI) is an important component of infections acquired from hospital. The most significant feature of vascular surgery different from other surgeries is frequent application of artificial grafts. Once SSI occurs after vascular operations with grafts, it might results in a serious disaster. *Staphylococcus aureus* and coagulase-negative *Staphylococcus* are the most common pathogenic bacteria for SSI after vascular surgery. Although SSI in vascular surgery often lacks of typical clinical characters, some clinical symptoms, laboratory data and certain imaging procedures may help to diagnose. In most cases of SSI after vascular procedures, the artificial grafts must be removed and sensitive antibiotics should be administered. However, for different cases, personalized management plan should be made depending on the severity and location of SSI.

## 1. INTRODUCTION

Vascular surgery is a new interdisciplinary subject of medicine. Besides has the general characteristics of other surgical disciplines, vascular surgery is characterized in that a variety of artificial graft (artificial blood vessels, stents, stent grafts) are widely used in clinical. Most vascular surgical operation is clean operation, but the chance of infection is usually increased, due to the application of artificial graft, and that vascular surgery patients are often elderly, and may be combined with a variety of internal medicine diseases such as diabetes, hypertension and heart disease, immune disease, weak body resistance. Once surgical site infection (SSI) is induced, the consequences would be disastrous. It’s not enough, sometimes, with antibiotic therapy alone for graft infection, and if necessary, removal of the infected vascular graft and revascularization pathway have to be operated [1-3], otherwise SSI can cause serious limb loss, organ failure, and even death.

## 2. RISK FACTORS

*Staphylococcus aureus* and coagulase-negative staphylococci are the most common pathogens of vascular surgery SSI. According to statistics, both early (within 4 months after operation) and late (more than 4 months after graft infection), one forth to a half risk is caused by *Staphylococcus aureus*, gram-negative bacteria, and fungal infections are rare, generally only occurs in immunosuppressed patients (Table **1**) [2].

The article "Diagnosis and Treatment of Vascular Surgery Related Infection" was retracted in 2018. Reason: compromised peer review.

### 2.1 Preoperative Pollution

The epidermis is the main source of bacteria. The graft surface can be contaminated by microbe through the following 3 ways: (1) Through transplantation of direct planting. An important way for the occurrence of the operation process of bacteria; and sweat glands, lymph node contact; graft and artery wall lesions connected; intestinal grafts or exudate pollution, exposure to injury or open gastrointestinal or genitourinary tract. (2) Through the operation incision. (3) By blood or lymphatic spread.

### 2.2 Bacteria Planting by Vascular Graft

The spread of bacteria by hematogenous pathway and planted in the graft or endovascular stent graft infection occurred is a common cause, but it is a very important mechanism. The animal experiments, perfused 10^7^ colony forming units (CFUs) of *Staphylococcus aureus*, experimental animal almost 100% in postoperative graft infection [3] occurred. In elderly patients with vascular disease, vascular catheter insertion, urinary tract infection or infection of the tissues (pneumonia or infected foot ulcer) often become the source of graft bacteria, and the occurrence of postoperative graft 

infection [3]. After several years of operation, when the change in the immune system, causing vascular graft infection exists in the blood can be contaminated bacteria. Some people think, possible mechanism of late graft infection: for transplantation when vascular surface pathogenic bacteria [4] dormancy.

### 2.3 Infection around Vascular Graft

Because of the skin, gastrointestinal or genitourinary tract pollution, vascular graft infection can be caused around.

## 3. DIAGNOSIS

### 3.1 Clinical Symptoms

Vascular graft infection is lack of typical clinical manifestations, such as aortic graft infection, may be manifested as unexplained bacteremia, or simply manifested as abdominal distension and muscle tension; lower extremity, groin or neck vascular transplantation, if graft infection can appear to invade surrounding tissue, vascular grafts exposed around the tumor, wound drainage sinus formation or pulsatile anastomotic aneurysm. In short, as long as there are no signs suggesting vascular graft infection, should be further examined.

### 3.2 Laboratory Tests

Once the vascular graft infection, the patient may have inflammation phenomenon of fever, white blood cell counts increased, erythrocyte sedimentation rate higher nonspecific (Fig **1**, Table **2**) [2, 3]. Routine laboratory tests should include analysis of urine and blood culture, and of any possible sources of infection bacteria. But the patient laboratory only two thirds positive results, and the vessel of Staphylococcus epidermidis delayed periallograft infection, all laboratory results can be negative.

The article "Diagnosis and Treatment of Vascular Surgery Related Infection" was retracted in 2018. Reason: compromised peer review.

### 3.3 Special Inspection Vessels

Using vascular ultrasound, CT and MRI, can be detected in vascular plants infected graft shift caused by the abscess or anastomotic aneurysm, selective joint use of such special vascular examination, diagnosis of vascular graft infection sensitivity can reach more than 80%, the specificity was 50% ~ 90%, and to help determine the surgical approach and the scope of 3; angiography in the planning of treatment has a guiding role; on suspicion of aortic graft infection patients must be two-way angiography, in order to understand the host and graft patency by the extent of infection and the proximal and distal vessels, in order to make further treatment.

## 4. TREATMENT

Without the use of artificial vascular surgical operation shift plant, the postoperative SSI treatment is same with other disciplines, including the principle of surgical debridement, washing, dressing and antibiotics when necessary. The use of artificial graft vascular surgical operation of plants, if SSI, has the special treatment, the standard surgical treatment plant blood vessel graft infection is: removal of the infected vascular graft, for extra anatomic bypass graft. But because of graft infection at different degree and scope, clinicians should according to the specific circumstances of vascular graft infection, to develop individualized treatment (Table **3**) [1].

### 4.1 Local Processing

Local treatment of plant blood vessel graft infection includes transplantation of vascular bed to infection fully debridement and drainage, need debridement, remove of purulent necrotic tissue, and the persistent aortic stump debridement treatment. Positive vascular graft is an effective local treatment of retained vascular grafts, reduce the basis of amputation. Through effective treatment, 70% cases can be successfully preserved vascular graft [5-8].

Vascular graft infection is widespread or involving the anastomosis, artificial blood vessels should be removed, both ends of the artery by single strand suture. Persistent aortic wall and surrounding tissues, especially in the presence of suppurative change or pseudoaneurysm arterial wall, should debridement to normal form artery, artery stump covered with sterile tissue with activity. Artery debridement must be used to confirm the histological examination, such as arterial wall bacterial cultures were positive, need long-term antibiotic therapy.

The removal of residual bed infection of vascular graft, thoroughly debridement, removal of necrotic tissue purulent, until the normal tissue exposure, the wound, the closed negative pressure drainage tube, do sufficient drainage.

The article "Diagnosis and Treatment of Vascular Surgery Related Infection" was retracted in 2018. Reason: compromised peer review.

### 4.2 Revascularization

The occurrence of vascular graft infection, limb collateral circulation only when fully established, only consider the simple removal of infected vascular grafts, without vascular reconstruction. But such cases are rare, usually removed vascular grafts were performed after revascularization. The general remove of the infected vascular graft, the need for extra anatomic bypass grafting, in order to save the organs and limbs. After removal of the infected graft, in situ with autogenous vein, artery allograft or antibiotic containing artificial blood vessel revascularization, extra anatomic bypass graft compared with more standard, simplify the operation process, shorten the operation time, improve the superiority and graft patency rate. But for in situ vascular transplantation, prone to infection and infection of retransplantation vascular anastomosis, so only without systemic infection, and perivascular per gram of tissue culture of less than 10^5^ units (CFUs), cloning is possible in situ transplantation of blood vessel [9-11]. Revascularization of transplanted autologous vascular material selection is the best, followed by artificial blood vessel, but in most cases not suitable for autologous vascular graft, can only use artificial blood vessels, through normal tissue without bacterial infection is consistent with the normal host artery (Fig. **2**) [1].

The general remove of the infected vascular graft, the need for extra anatomic bypass, in order to save the organs and limbs. The following is the classification of treatment according to different parts of the vascular graft infection.

#### 4.2.1 Aortic, Iliac Artery Vascular Graft Infection

The aorta and iliac artery vascular graft infection, the most reasonable treatment principle is: first the right axillary artery to bilateral femoral artery bypass surgery; complete dissection, with sterile dressings covering all the wounds, and then open the complete removal of vascular graft infection. In extra anatomic revascularization, should be heparin therapy; artificial blood vessel and remove the infection, with heparin antagonists.

The extra anatomic bypass surgery and postoperative complications, statistical data shows that: the operation mortality was 11% ~ 27%, the amputation rate occurred as 9%~27% [12,13], so as to have allogeneic vascular grafts, may be considered for in situ revascularization, can significantly reduce postoperative complications. But most of the medical institutions are unconditional access to these vessels.

#### 4.2.2 Aorta Bilateral Femoral Artery Vascular Graft Infection

Aorta bilateral femoral artery graft infection treatment is difficult, because the inguinal region of vascular graft infection, affect the lower limb blood supply, for extra anatomic bypass reconstruction, the distal anastomosis should be built in the deep femoral artery or superficial femoral artery to artery, even, in order to avoid the occurrence of lower extremity ischemic necrosis. The graft should choose diameter greater than 5mm or PTFE artificial blood vessels of saphenous vein.

The article "Diagnosis and Treatment of Vascular Surgery Related Infection" was retracted in 2018. Reason: compromised peer review.

Occurred in the late postoperative and localized in the inguinal region of vascular graft infection, can be considered part of the partial resection of the infected vessels, after thorough debridement, in situ revascularization; postoperative intravenous antibiotics for 2~4 weeks, and continued to take 3 months.

#### 4.2.3 Femoral and Tibial Artery Vascular Graft Infection

Inguinales artificial vascular bypass vascular graft infection, are generally required to remove the artificial blood vessel. The treatment should follow the principle of treatment of vascular aortic graft infection, although the mortality rate is low, but the possibility of amputation is higher than 50% [14-17].

Such as the removal of the infected vessels, ankle arterial pressure or forearm pressure greater than 40mmHg (1mmHg = 0.133kPa), suggesting that body can delay the establishment of collateral circulation, graft revascularization, and anti-inflammatory treatment, control of infection after revascularization, again to increase vascular grafting patency rate, reduce complications.

#### 4.2.4 Innominate Artery, Subclavian Artery and Carotid Artery Vascular Graft Infection

Intrathoracic vascular graft infection, the treatment principle is: to remove the entire graft, vascular reconstruction with autologous vascular graft materials as much as possible, and intravenous injection of antibiotics. The remove of grafts, in order to control the proximal vessels, often require incision and median clavicle, cardiopulmonary bypass.

Because the upper limb ischemia underwent transthoracic or extrathoracic bypass surgery, and the occurrence of vascular graft infection, resection of the infected vascular graft, generally do not need immediate revascularization; because the upper limb necrosis due to ischemia and rarely occur. Re revascularization in complete control after infection, and can increase the success rate of transplantation operation.

Carotid artery bypass vascular graft infection, artery ligation in general can’t tolerate simple, only when the carotid stump pressure is greater than 70mmHg, it can only simple ligation of common carotid artery and internal carotid artery [18]. But in order to ensure the blood perfusion of cerebral circulation, prevent the occurrence of shock, it should be possible for revascularization.

The article "Diagnosis and Treatment of Vascular Surgery Related Infection" was retracted in 2018. Reason: compromised peer review.

Carotid endarterectomy artificial patch infection, should be artificial patch resection of the carotid artery, using autologous vascular patch, in the process of operation, the carotid artery bypass is safe and effective measures of cerebral blood flow.

#### 4.2.5 Stents and Endovascular Infection

The endovascular exclusion in the surgical trauma, the intestinal tract and other organs significantly reduce interference, shorten the operation time, intraoperative and postoperative blood transfusion without the above factors, significantly reduce the chance of graft infection. Therefore, intraluminal vascular graft infections are more rare. But the endoscopic operation of complex technology and instruments are more numerous, the need for surgery in the DSA, so as to increase the chance of graft infection. Once the endovascular graft infection, often associated with sepsis and infection of the aneurysm and thrombus shedding bacteria, the most common pathogenic bacteria were *Staphylococcus aureus*, artery plants and infection involving the shift treatment including removal of the cavity, parallel extra anatomic bypass, according to different parts of the vascular graft infection. Select the vascular reconstruction schemes of different [19].

## CONCLUSION

Antibiotic-loaded PMMA beads may serve as an adjunct in the management of VSSIs and may also expand treatment options for graft preservation or in situ reconstruction, with expected recurrent infection rate approaching 20%. Further experience with this adjunct may help elucidate its role in the management of this complicated problem, including the need for bead exchanges, until perigraft cultures are free of microbes.

## Figures and Tables

**Fig. (1):** Scatterplot of total bacterial counts (colony-forming units /mL) in patients with and without surgical site infection (y-axis in log10scale). Note. SSI = surgical site infection.

**Fig. (2):** Comparison of time to treatment failure in different types of prosthetic vascular graft infections. infections are compared with respect to the location of the prosthetic vascular graft using kaplan-meier estimates.

**Table 1.** Binary logistic regression analysisa of factors associ-ated with surgical wound infection after lower limb vascular surgery.

Risk factor	OR	95% CI	p
CFU/mL >155,000 on the second postoperative day	5.97	1.67–21.42	.006
Diabetes	4.77	1.46–15.55	.010
Elective redo surgery	0.16	0.03–0.88	.035
Infra-inguinal surgery	4.11	0.95–17.84	.059
Male gender	4.41	0.90–21.71	.068

Note. OR = odds ratio; CI = confidence interval; CFU = colony-forming unit. ^a^ Regression model with CFU/mL >155,000 on the second postoperative day, diabetes, elective redo surgery, infra-inguinal surgery, and sex as covariates.

The article "Diagnosis and Treatment of Vascular Surgery Related Infection" was retracted in 2018. Reason: compromised peer review.

**Table 2.** Type and number of bacterial and fungal isolates recovered from 42 vascular surgical sites.

Type	No.
Gram-positive	
Staphylococcus aureus	
Methicillin-resistant	10
Methicillin-sensitive	5
S. epidermidis	6
Enterococcus	7
Streptococcus spp	2
Methicillin-resistant S. epidermidis	1
Vancomycin-resistant Enterococcus	1
Bacteroides spp	7
Total	39
Gram-negative	
Escherichia coli	7
Pseudomonas	3
Haemophilus	1
Proteus	1
Citrobacter	1
Klebsiella	1
Enterobacter	2
Propionibacterium acnes	2
Total	18
Candida	2
No growth	2

**Table 3.** Predictors of cure at one year in 51 patients with aortic prosthetic vascular graft infections.

Variable	Univariate Analysis			Multivariate Analysis		
	HR	95% CI	p-Value	HR	95% CI	p-Value
Age	0.33	0.15–0.74	0.007	0.45	0.19–1.11	0.083
Female gender	0.96	0.15–6.35	0.970	—	—	—
Location of the Graft						
Thoracic	1	—	—	—	—	—
Abdominal, with noiliac-femoral graft involvement	0.14	0.02–1.06	0.057	—	—	—
Abdominal withiliac-femoral graft involvement	0.07	0.02–0.32	0.001	0.24	0.05–1.16	0.076
Intubation >24 hours	0.44	0.10–1.91	0.276	—	—	—
Early surgical graft revision <24 hours after implantation	1.30	0.42–4.03	0.645	—	—	—
Polymicrobial infection	0.72	0.23–2.24	0.573	1.93	0.41–9.13	0.405
Type of Surgical Treatment						
Graft retention and debridement	0.46	0.14–1.50	0.196	—	—	—
Graft replacement	0.87	0.23–3.26	0.842	0.89	0.15–5.31	0.899
Local Surgical Therapy Associated with Graft Revisions/Replacements						
Vacuum-assisted closure	0.54	0.16–1.88	0.335	—	—	—
Plastic surgery	0.96	0.15–6.35	0.970	—	—	—
Antimicrobial Therapy						
Antimicrobial regimen that included rifampicin	7.85	1.90–32.4	0.004	6.88	1.33–35.4	0.021
